# Iopromide and Iodixanol in the Development of Postoperative Contrast Nephropathy in Patients with Renal Insufficiency: A Meta-Analysis

**DOI:** 10.1155/2022/1469370

**Published:** 2022-04-05

**Authors:** Yiyu Feng, Guoping Qiu, Chengyun Xu, Zhibing Duan, Manting Wang, Lamei Wang, Wenjie Hu, Peifang Li, Hui Zhou

**Affiliations:** ^1^Department of Nephrology, Jiujiang First People's Hospital, Jiujiang 332000, China; ^2^Department of Nephrology, The Second Affiliated Hospital of Nanchang University, Nanchang 330000, China; ^3^Department of Nephrology, Nanchang Third Hospital, Nanchang 330000, China

## Abstract

In order to compare the effects of iopromide and isoxazole on postoperative contrast-induced nephropathy in patients with renal insufficiency, the paper searches for randomized controlled trials and retrospective cohort studies comparing the effects of iopromide and iodixanol on renal function in patients with renal insufficiency after surgery. The data are extracted from eligible studies. We tried to assess the incidence of contrast-agent nephropathy, preoperative and postoperative serum creatinine indicators, and mortality. This paper includes 8 studies with a total of 1243 patients. The incidence of contrast-induced nephropathy in the iopromide group is higher than that in the iodixanol group, and there is no significant difference between the two groups in postoperative mortality and preoperative serum creatinine expression. Sensitivity analysis and funnel chart show that our research is robust and has low publication bias. Our research shows that in patients with renal insufficiency, the incidence of contrast-medium nephropathy in the iopromide group is higher than that in the iodixanol group. Iodixanol is safer and has less effect on patients' serum creatinine levels.

## 1. Introduction

With the continuous advancement of medical technology, interventional diagnosis and treatment technology have been widely used in clinical practice, and the use of contrast agents has also increased. Although the development of medical technology has made the adverse reactions of contrast agents less and less, there are still some patients who experience heart disease in clinical practice [1, 2], renal insufficiency, and even death of the patient. A contrast agent is excreted through the kidneys, which has a more significant impact on renal function, mainly when patients over 70 years of age use contrast agents for coronary intervention surgery [3–5]. The probability of contrast agent nephropathy is greater. Therefore, clinically selecting a reasonable contrast agent is of great significance to reduce renal function damage [6–8].

Iopromide is a new, nonionic, hypotonic contrast agent. Suitable for CT enhanced scan, digital silhouette angiography (DSA), intravenous urography, extremity angiography (including arterial and venography), and body cavity angiography (including arthrography, hysterosalpingography, sinus angiography, but not for arachnoid Inferior cavity angiography, ventricle cisternography) [9–11].

Iodixanol is a nonionic isotonic contrast agent, which will not affect the secretion of renal tubular enzymes and glomerular filtration function, even if it has a minimal effect. Iodixanol has low osmotic pressure and causes minor local irritation to patients [12, 13]. During the treatment, the patient feels less pain and can maintain the position required for the operation for a long time under local anesthesia.

Contrast-induced nephropathy (CIN) is a common complication of coronary intervention. It is caused by the use of iodine contrast agents [14–16]. The overall incidence rate in the population is 2% to 3% E-1, but in patients with high-risk factors such as advanced age, chronic renal insufficiency, diabetes, and congestive heart failure, it is much higher. The incidence of CIN is 20% to 30%. Therefore, we conducted this meta-analysis.

## 2. The Proposed Scheme

### 2.1. Literature Search Strategy

Seven electronic databases, including PubMed, EMBASE, Cochrane Library, CBM, CNKI, Wan fang, and Chinese science, have established VIP to search systematically from 2002 to 2021. We used the following keywords: iopromide; (2) isoxazole; (3) renal insufficiency; and (4) contrast nephropathy. A Boolean-search strategy is used with the operators “AND,” “NOT,” and “OR” as well as paper keywords related to physical fitness, PET. A comprehensive search of the literature is performed without restricting languages, publication date, or publication status. Two individual reviewers identified and reviewed full-text articles and abstracts deemed relevant by screening the list of titles. Disagreements between the two reviewers are resolved with consensus.

### 2.2. Paper Selection

After the preliminary selection of studies, the relevant research texts should be reviewed. The included studies must meet the following inclusion criteria: (1) the subjects are patients with renal insufficiency; (2) iopromide and iodixanol are compared; (3) the incidence of contrast-induced nephropathy; and (4) the full text is available. Non-RCTs, nonhuman studies, conference abstracts and summaries, and reviews or meta-analyses are excluded from consideration. We excluded patients with diabetes, renal transplants, and hypersensitivity to iodides because they confuse treatment outcomes. Studies published only as abstracts are included after the authors are contacted for more detailed information. If multiple publications from the same queue are available, we extract data from the largest or most recent dataset.

### 2.3. Data Extraction and Quality Assessment

The studies are reviewed and the data are extracted independently by two of the investigators. The following information is extracted from the registered article: (1) name of the first author, (2) year of publication, (3) country of origin, (4) sample size, (5) age (and gender) of the sample, and (6) paper duration. We made critical assessments separately for each domain. We graded it as low risk for bias, unclear risk, or high risk for bias according to the criteria specified in the Cochrane Handbook.

### 2.4. Statistical Analysis

The Review Manager (version 5.2, Cochrane Collaboration, 2011) is used to estimate the impact of the results in the selected report. The between-paper heterogeneity is assessed using Cochran's Q statistic and quantified by the *I*^2^ statistic. We considered *I*^2^ values ≥50% to indicate substantial heterogeneity and values ≥75% considerable heterogeneity. Heterogeneity between and within designs is assessed using Cochran's Q and quantified using *I*^2^ statistics. *I*^2^ values of less than 25%, 25% to 75%, and greater than 75% represented low, moderate, and high degrees of heterogeneity, respectively.

The random-effect model is applied if the heterogeneity is observed, whereas the fixed-effect model is involved in the absence of between-paper heterogeneity. Publication bias is represented graphically by funnel plots of the standard difference in means versus the standard error. A visual inspection of funnel plot asymmetry is performed to address the possible small-paper effects. A sensitivity analysis was further conducted to evaluate the robustness of the findings through exponential tilting.

## 3. The Experimental Results

### 3.1. Search Process

A total of 942 articles were identified in this search, with a further fifty identified following a review of references of other reports. After removing duplicates, 752 records remained. By screening the titles and abstracts, an additional 163 records are excluded because they are review articles, letters, case reports, comments, or editorials. In consideration of the paper design and insufficient data presented, 52 articles are rejected. Ultimately, eight studies that met the selection criteria are included in the present meta-analysis. The results of the search process are illustrated in a flowchart, as shown in Figure 1.

### 3.2. Characteristics of Included Studies

Table 1 shows the main characteristics of the included studies, including 1243 patients with renal insufficiency. Of the 1243 participants, 684 (55%) were male. The average age is 55–81 years old. The primary outcome measures are the incidence of CIN, the comparison of serum creatinine levels before and after treatment, and mortality. All eight articles were published from 2003 to 2019. A total of 1243 patients with renal insufficiency were included in these studies, 642 in the iopromide group and 601 in the iodixanol group.

### 3.3. Results of Quality Assessment

The Cochrane risk of bias assessment tool is used to evaluate the risk of included studies. The quality of studies included in the review is evaluated by two independent reviewers, with differences resolved by consensus or through a third reviewer if required.  Figure 2 shows risk of bias of included studies: low (green), unclear (yellow), and high (red). A summary of all kinds of bias in each paper is shown in Figure 3. In general, there are two trials with a bias risk, and six trials have no risk.

### 3.4. Results of Heterogeneity Test

We use a meta-analysis based on a fixed-effects model to calculate the average difference. The overall average difference is 0.71, and the 95% confidence interval is 0.35, 1.43. The overall curative effect *P* value = 0.02, *I*^2^ = 65%, indicating that there is a significant difference in the probability of contrast nephropathy between the iopromide group and the iodixanol group.  Figure 4 shows that the iopromide group is significantly more than the iodixanol group.

We conducted a meta-analysis of the mortality of patients in the iodixanol group and iopromide group after adjuvant treatment. The results showed that there is no significant difference in postoperative mortality between the two groups (OR = 0.31, 95% CI [0.06, 1.16], *P*=0.98; fixed-effect model).  Figure 5 shows a forest chart: a comparison of postoperative mortality between two groups.

Heterogeneity analysis of preoperative serum creatinine levels in the iopromide group and iodixanol group is reported in four studies involving 471 patients. Meta-analysis showed that there is no significant difference in serum creatinine level between the two groups (MD = −1.09, 95% CI [−7.37, 5.19], *P*=0.12; random effect model), and the heterogeneity is not significant (*i*^2^ = 49%).  Figure 6 shows forest map: a comparison of preoperative serum creatinine levels between the two groups.

Heterogeneity analysis of postoperative serum creatinine levels in the iopromide group and iodixanol group is reported in four studies involving 471 patients. Meta-analysis showed that there is significant difference in serum creatinine level between the two groups (MD = −2.8, 95% CI [−21.26, 15.66], *P*=0.010; random effect model), and the heterogeneity is significant (*i*^2^ = 74%).  Figure 7 shows a forest map: comparison of serum creatinine levels between two groups after operation.

### 3.5. Results of Sensitivity Analysis and Publication Bias

A total of five studies reported the incidence of contrast-induced nephropathy after surgery. The forest map showed that the incidence of the iopromide group is higher than that of the iodixanol group (or = 0.71, 95% CI [0.35, 1.43], *P*=0.02, i.e ^2^ = 65%; Figure 4). We conducted a sensitivity analysis by removing Shin 2011, and the results showed little change. The change from 65% to 63% (Figure 8) indicates that the results of the included articles are robust.

We also plotted a funnel plot to assess publication bias in the incidence of contrast-induced nephropathy. The figure shows that the shape is not symmetrical. This indicates that there is little publication bias in this meta-analysis. Figure 8 shows a sensitivity analysis of the incidence of contrast-induced nephropathy in two groups.  Figure 9 shows a funnel plot showing publication bias.

## 4. Experimental Result and Discussion

Our paper showed that the incidence of contrast-induced nephropathy in the iopromide group is higher than that in the iodixanol group, and there is no significant difference in preoperative serum creatinine level between the two groups (*P* > 0.05). The serum creatinine level of the two groups after the operation is higher than that before the operation, and the iopromide group is higher than that of the iodixanol group. The difference is statistically significant (*P* < 0.05). Lu's research shows that in elderly patients with renal insufficiency, it is safer to use iodixanol as a contrast agent in coronary interventional surgery and has a negligible effect on the serum creatinine level of patients. It can reduce the incidence of contrast-induced nephropathy and is worthy of widespread clinical application.

## 5. Conclusion

Studies have shown that with the development of modern imaging technology, contrast-induced nephropathy (CIN) has been paid more and more attention by nephrologists, can refer to the sudden decrease of renal function caused by contrast medium. The commonly used contrast agent is hypertonic, and the iodine content is as high as 37%. They are filtered by the glomeruli in the body and are not absorbed by the tubules. Dehydration, the concentration of drugs in the kidney increases, will cause kidney damage. Acute renal failure occurred. Iodixanol is an isotonic nonionic contrast agent. It is mainly an iodine-containing contrast agent, which is primarily used for diagnosis and medication in cerebrovascular angiography, peripheral arteriography, abdominal angiography, and urography interventional therapy.

The paper also has some limitations. For example, the data of this paper did not include the data of complications and controlled trials in young patients. In addition, due to the limitation of the quantity and quality of the paper, it needs to be confirmed by a large-sample, multicenter follow-up controlled trial.

## Figures and Tables

**Figure 1:** Flowchart of the literature search and paper selection.

**Figure 2:** Risk of bias of included studies: low (green), unclear (yellow), and high (red).

**Figure 3:** Risk of bias summary.

**Figure 4:** Forest chart: comparison of the incidence of contrast-induced nephropathy between the two groups.

**Figure 5:** Forest chart: a comparison of postoperative mortality between two groups.

**Figure 6:** Forest map: comparison of preoperative serum creatinine levels between the two groups.

**Figure 7:** Forest map: a comparison of serum creatinine levels between two groups after operation.

**Figure 8:** Sensitivity analysis of the incidence of contrast-induced nephropathy in two groups.

**Figure 9:** Funnel plot showing publication bias.

**Table 1:** Clinical baseline information of all the included patients.

Paper	Year	Language	Country	Groups	Sex (male/female)	Age (years)	Patients (*n*)	Years of onset
Gao	2020	Chinese	China	Iodixanol	21/14	66.5 ± 8.37	35	2017 to 2019
				Iopromide	23/12	70.75 ± 4.62	35	
Hsieh	2006	English	China	Iodixanol	17/10	73 ± 1	27	2004 to 2005
				Iopromide	23/4	71 ± 1	27	
Juergens	2009	English	Australia	Iodixanol	72/19	70.2 ± 9.2	91	2003 to 2006
				Iopromide	73/27	69.4 ± 10.2	100	
Nie	2008	English	China	Iodixanol	73/33	61 ± 11.5	106	2005 to 2006
				Iopromide	69/33	60 ± 12.3	102	
Qian	2017	English	China	Iodixanol	36/9	63 ± 13	45	2015 to 2015
				Iopromide	32/13	62 ± 13	45	
Shin	2011	English	Korea	Iodixanol	110/105	71.1 ± 8.7	215	2009 to 2010
				Iopromide	116/89	71.9 ± 8.2	205	
Wen	2018	Chinese	China	Iodixanol	28/14	79.63 ± 3.25	42	2015 to 2016
				Iopromide	29/13	79.89 ± 3.68	42	
Zheng	2010	Chinese	China	Iodixanol	28/12	71 ± 8	40	2004 to 2009
				Iopromide	61/25	70 ± 8	86	

## Data Availability

The simulation experiment data used to support the findings of this study are available from the corresponding author upon request.
